# The Effect of FRAX on the Prediction of Osteoporotic Fractures in Urban Middle-aged and Elderly Healthy Chinese Adults

**DOI:** 10.6061/clinics/2017(05)06

**Published:** 2017-05

**Authors:** Jun Wang, Xuejun Wang, Zhen Fang, Nanjia Lu, Liyuan Han

**Affiliations:** I Director’s Office, Minglou Street Community Health Service Center, Jiangdong District, Ningbo, China; II Director’s Office, Dongliu Street Community Health Service Center, Jiangdong District, Ningbo, China; III Department of Preventive Medicine, Zhejiang Provincial Key Laboratory of Pathophysiology, School of Medicine, Ningbo University, Ningbo, China

**Keywords:** FRAX, Osteoporotic Fracture, Bone Mineral Density

## Abstract

**OBJECTIVE:**

We aimed to analyze the applicability of a fracture risk assessment tool for the prediction of osteoporotic fractures in middle-aged and elderly healthy Chinese adults.

**METHODS:**

A standard questionnaire was administered, and bone mineral density was measured in residents visiting the Dongliu Street Community Health Service Center. Paired t-tests were used to compare the FRAX-based probabilities of fractures estimated with and without consideration of bone mineral density. Risk stratification and partial correlation analyses were applied to analyze the associations between FRAX-based probabilities and body mass index or bone mineral density at different sites.

**RESULTS:**

A total of 444 subjects were included in this study. Of these subjects, 175 (39.59%) were diagnosed as osteoporotic, and 208 (47.06%) were diagnosed as osteopenic. The Kappa value for the detection of osteoporosis at the L1-L4 lumbar spine and femoral neck was 0.314. The FRAX-based 10-year major osteoporotic fracture probability and hip osteoporotic fracture probability estimated without considering bone mineral density were 4.93% and 1.64%, respectively; when estimated while considering bone mineral density, these probabilities were 4.97% and 1.54%, respectively. A significant positive association was observed between the FRAX-based fracture probabilities estimated with and without consideration of bone mineral density, while significant negative associations between body mass index and the estimated FRAX-based fracture probabilities after adjustment for age and the estimated FRAX-based fracture probabilities and femoral neck bone mineral density were identified. These results remained the same after controlling for lumbar spine bone mineral density.

**CONCLUSIONS:**

The Chinese FRAX model could predict osteoporotic fracture risk regardless of whether bone mineral density was considered and was especially appropriate for predicting osteoporotic fractures of the femoral neck.

## INTRODUCTION

Osteoporotic fractures are important causes of morbidity and place a heavy burden on China’s healthcare system 1. Bone mineral density (BMD), as detected by dual-energy X-ray absorptiometry (DXA), is an accepted diagnostic index for osteoporosis; however, DXA is very expensive and has not been widely applied in primary health care settings in China. A fracture risk assessment tool (FRAX) has been developed by the World Health Organization (WHO) 2. By considering age, gender, BMD, body mass index (BMI), and other easily obtainable risk factors, the FRAX model can assess a patient’s 10-year major osteoporotic fracture probability (MOFP) and 10-year hip osteoporotic fracture probability (HOFP) 2. FRAX has been successfully used in the UK 3, the USA^4^ and Poland 5. A French study found that the estimated FRAX-based 10-year osteoporotic fracture probability was lower than the actual observed fracture rate in women with low BMD who were over 65 years of age 6; similar results were also observed in a prospective cohort study performed in Spain 7.

Due to contextual differences between countries, the FRAX model should be calibrated based on each country’s own epidemiologic data 8,9. The thresholds for therapeutic intervention in postmenopausal women in South-central China 10 are lower than those in the UK 3, Hong Kong 11, and Sri Lanka 8. Therefore, we applied the FRAX model in a population of middle-aged and elderly healthy (without current serious diseases) community residents to evaluate the fracture probabilities at different sites and assess the applicability of FRAX in Ningbo, China. The prevalence rate of osteoporosis in Ningbo, which is a coastal city in Eastern China with frequent rainstorms and typhoons, observed in those below the age of 60 years is higher than the prevalence rates reported in other regions in China 1,14, and data suggest that the peak BMD is lower and osteoporosis occurs earlier in residents of Ningbo than in residents of other areas in China 12,13.

## METHODS

### Study subjects

Subjects were consecutively enrolled between July 2013 and June 2015 from the Dongliu Street Community Health Service Center in Ningbo, China. We applied a simple random procedure according to a sequence of computer-generated random numbers to recruit eligible subjects. The inclusion criteria were as follows: healthy subjects aged between 40 and 89 years, healthy local permanent residents who had lived in Ningbo since birth, healthy subjects without a diagnosis of osteoporosis and not taking some certain related drugs, and subjects who could participate in the study independently. All study subjects provided written informed consent, and the study was approved by the Medical Ethics Committee of Jiangdong District. A questionnaire including sociodemographic factors, chronic disease history, menstruation and reproductive history, lifestyle factors, dietary habits and other osteoporosis-related factors was completed by all subjects with the help of trained assistants. A comprehensive physical examination (including BMD, height, weight, electrocardiography and routine blood tests) was also performed.

### FRAX calculation

The 10-year MOFP (hip, clinical spine, humerus or wrist fracture) and the 10-year HOFP were computed using the FRAX model (http://www.shef.ac.uk/FRAX) 15. Fracture risk was calculated based on age, BMI and dichotomized risk factors (comprising prior fragility fractures, parental history of hip fractures, smoking, alcohol consumption, history of steroid use, rheumatoid arthritis and other causes of secondary osteoporosis). In addition, we entered the femoral neck (FN) BMD into the model to enhance its ability to predict fracture risk 16.

### BMD evaluation

BMD was detected at the L1-L4 lumbar spine (LS), FN, and total hip using DXA (Lunar Prodigy, GE, USA). The DXA results were adjusted for age and weight, and Chinese adults aged 20-40 years were used as the reference group. All BMD measurements were performed by a trained licensed technologist. A T score≤-2.5 indicated osteoporosis, a T score>-2.5 and ≤-1.0 indicated osteopenia, and a T score>-1.0 indicated normal BMD^1^.

### Statistical analysis

Quantitative data are presented as the mean±standard deviation (SD) and were analyzed using Student’s t-tests or one-way ANOVA. Qualitative data are expressed as numbers (percentages) and were analyzed using chi-squared tests. Paired t-tests were used to compare the probabilities of fracture estimated with and without consideration of BMD. Risk stratification and partial correlation analyses were used to analyze the associations between FRAX-based probabilities and BMI or BMD at different sites. P-values<0.05 were considered statistically significant. All statistical analyses were performed using SPSS version 13.0 (SPSS, Chicago, IL).

## RESULTS

### Basic characteristics and FRAX-based osteoporotic fracture probability

A total of 444 (80 males/364 females) subjects were included in this study, and 98% of female subjects were postmenopausal women. Statistically significant differences were found for age, current smoking, current alcohol consumption and secondary osteoporosis between male and female subjects (Table 1). Of the subjects, 175 (39.59%) were diagnosed as osteoporotic, and 208 (47.06%) were diagnosed as osteopenic (Table 1). The rate of osteoporosis was significantly higher among females than males. The Kappa value for the detection of osteoporosis at the LS and FN was 0.314. Statistically significant differences were observed between males and females for the FRAX-based 10-year MOFP and HOFP estimated without consideration of BMD and the 10-year MOFP estimated with consideration of BMD (Table 1). The MOFP and HOFP estimated with and without the consideration of BMD increased with age (Table 2). Significant positive associations were observed between the HOFPs estimated with and without consideration of BMD (r=0.761, P<0.001) and the MOFPs estimated with and without consideration of BMD (r=0.804, P<0.001); however, no significant differences were observed subjects with and subjects without BMD measurement.

### The association between FRAX-based fracture probability and BMI

Significant negative associations were observed between BMI and FRAX-based fracture probabilities after adjusting for age among the overall subjects, and this difference was especially significant in males and in females when FRAX-based probabilities were calculated without consideration of BMD. While FRAX-based probabilities were calculated with consideration of BMD, a significant association between fracture probability and BMI was only identified in females (Table 3)</underline>.

### FRAX-based fracture probabilities among subjects with different BMD levels

Among the three BMD groups (osteoporotic, osteopenic and normal BMD), FRAX-based fracture probabilities were highest in the osteoporosis group and lowest in the normal BMD group. This result remained the same regardless of the diagnostic standards applied. However, in our risk stratification analyses, we found that the estimated FRAX-based fracture probabilities were primarily associated with FN BMD instead of LS BMD. When three stratums were classified based on FN BMD, and then three groups were classified based on LS BMD within each stratum, no statistically significant differences were found among the three groups within each stratum (Table 4). When three stratums were classified based on LS BMD, and then three groups were classified based on FN BMD within each stratum, statistically significant differences were observed among the three groups within each stratum (Table 4). Moreover, significant negative associations were found between the estimated FRAX-based fracture probabilities and FN BMD, even after controlling for LS BMD. Significant negative associations were also observed between the estimated FRAX-based fracture probabilities and LS BMD; however, these significant associations did not remain after controlling for FN BMD (Table 5).

## DISCUSSION

In this study, 39.59% of middle-aged and elderly healthy subjects in Ningbo (24.05% males and 42.80% females) were diagnosed as osteoporotic, and these detection rates were higher than the rates previously detected among residents aged over 50 years in China (14.4% males and 20.7% females) 1. The FRAX-based fracture probabilities (MOFP 4.93%, HOFP 1.64%) identified in this study were higher than the fracture probabilities previously reported in China, such as the probabilities reported in postmenopausal women in Beijing (MOFP of 2% to 4%, HOFP of 0.2% to 1.6%) 17. Additionally, the fracture probabilities identified in this study were much lower than those previously reported in Taiwanese postmenopausal women (MOFP 13.8%, HOFP 2.2%) 18, postmenopausal women in Hong Kong (MOFP 6.9%, HOFP 2.3%) 11, healthy subjects in the US 3, and women aged ≥50 years in Canada 9.

In this study, the major fracture rate was 2.48% after 1 year of follow-up. Ba et al. found that when the FRAX-based 10-year MOFP was greater than 3% or the HOFP was greater than 1%, the fracture rates at any site were 13.04% among subjects who had received treatment and 31.58% among subjects who had not received any treatment after 2 years of follow-up 19. Furthermore, consistent with the review conducted by Zhang et al. 20 and the research performed by Min et al. 21, we believe the FRAX model may underestimate the actual fracture probability in China.

Consistent with the study conducted by Fujiwara et al. 22, the FRAX-based fracture probability identified in females was significantly higher than that identified in males in this study, and these results remained stable in different age groups. We found a significant positive association between the FRAX-based osteoporotic fracture probabilities estimated with and without the consideration of BMD, which were both significantly associated with BMD. Similar results were reported in studies conducted in Korea 23 and Beijing 17, and the authors of these studies suggested that the FRAX-based osteoporotic fracture probabilities without and with consideration of BMD could predict the risk of fracture.

Interestingly, we found that the estimated FRAX-based osteoporotic fracture probabilities were strongly associated with FN BMD, especially when BMD was not considered. Risk stratification and partial correlation analyses did not indicate significant associations between the estimated FRAX-based osteoporotic fracture probabilities and LS BMD. Based on these results, it may be inferred that the FRAX tool is more appropriate for the prediction of the osteoporotic fracture of the FN than for osteoporotic fractures of the LS.

Notably, we identified significant negative associations between BMI and FRAX-based fracture probabilities estimated without consideration of BMD. This association was especially significant in subjects with a BMI less than 19, who have an obviously higher fracture risk; however, for subjects with a BMI greater than 19, the fracture risk remained relatively stable. This result was similar to those reported by other studies 24,25, suggesting that the relationship between BMI and FRAX-based fracture probability is nonlinear and that a low BMI (<19) might be a risk factor for fracture.

Our study has limitations. The sample size was relatively small; therefore, the extrapolation of our results to the whole population should be performed with caution. The FRAX-based fracture probabilities identified in our study could not be well-verified based on actual fracture rates because the follow-up period of our study was not sufficiently long to obtain sufficient fracture data. Therefore, our results require further confirmation, which we intend to perform in a future study. Nevertheless, our study validates the applicability of the FRAX model in Ningbo, a coastal city in Eastern China with a high prevalence of osteoporosis.

In conclusion, osteoporosis imposes a heavy burden on the population in Ningbo. The Chinese FRAX model could predict osteoporotic fracture risk regardless of whether BMD was considered. This model may be useful to predict osteoporotic fractures of the FN but has a limited ability to predict osteoporotic fractures of the LS. As the Chinese FRAX model may underestimate osteoporotic fracture risk, larger cohort studies that determine actual fracture rates are needed to validate and adjust the Chinese FRAX model. However, the FRAX model may have substantial value for screening and identifying those with a higher risk of osteoporotic fractures in China, especially in many primary medical facilities where BMD cannot be tested due to a lack of DXA equipment.

## AUTHOR CONTRIBUTIONS

Wang J assisted with the data collection, protocol development and manuscript preparation. Wang X, Fang Z and Lu N contrib ted to the protocol development and manuscript preparation. Han L contributed to the data collection, protocol development, s atistical analysis and manuscript preparation. All authors read and approved the final version of the manuscript.

## Figures and Tables

**Table 1:** Basic characteristics and FRAX-based 10-year osteoporotic fracture probabilities.

	Total	Males	Females	χ^2^ or t	P
Age	63.18±8.93	66.31±8.38	62.49±8.91	3.514	<0.001
BMI^1^	23.72±3.15	24.60±3.23	23.53±3.10	2.783	0.006
BMI<18.5	21 (4.73%)	4 (5.00%)	17 (4.67%)	0.015	0.904
Prior fracture	99 (22.30%)	20 (25.00%)	79 (21.70%)	0.857	0.602
Parental history of fracture	46 (10.36%)	8 (10.00%)	38 (10.44%)	0.014	0.907
Current smoking	19 (4.28%)	16 (20.00%)	3 (0.82%)	54.288	<0.001
Current alcohol consumption	46 (10.36%)	29 (36.25%)	17 (4.67%)	70.429	<0.001
History of steroid use	11 (2.48%)	2 (2.50%)	9 (2.47%)	<0.001	0.989
Rheumatoid arthritis	21 (4.73%)	1 (1.25%)	20 (5.49%)	1.765	0.184
Secondary osteoporosis	34 (7.66%)	1 (1.25%)	33 (9.07%)	5.666	0.017
Osteoporosis	175 (39.59%)	19 (24.05%)	156 (42.98%)	9.725	0.008
Osteopenia	208 (47.06%)	47 (59.49%)	161 (44.35%)		
MOFP^2^ without BMD^3^	4.93±3.30	3.41±1.77	5.26±3.46	6.859	<0.001
HOFP^4^ without BMD^3^	1.64±1.90	1.32±1.25	1.71±2.01	2.227	0.027
MOFP^2^ with BMD^3^	4.97±3.53	3.75±2.17	5.24±3.71	4.746	<0.001
HOFP^4^ with BMD^3^	1.54±2.21	1.53±1.64	1.55±2.32	0.093	0.926

1 BMI: body mass index;

2 MOFP: the FRAX-based 10-year major osteoporotic fracture probability;

3 BMD: bone mineral density;

4 HOFP: the FRAX-based 10-year hip osteoporotic fracture probability.

**Table 2:** FRAX-based 10-year osteoporotic fracture probabilities among subjects in different age groups.

Age (years)	N	Without BMD^1^		With BMD	
		Major fracture	Hip fracture	Major fracture	Hip fracture
<50	22	1.78±0.74	0.20±0.18	1.90±0.48	0.28±0.26
50-59	133	3.37±2.13	0.58±0.60	3.59±2.12	0.67±0.79
60-69	191	5.32±3.20	1.61±1.69	5.44±3.80	1.55±2.44
70-79	79	6.40±3.41	3.08±2.18	6.31±3.84	2.89±2.66
≥80	19	9.34±3.92	4.96±2.02	7.41±3.73	3.28±1.72
Variance test F		31.439	58.676	16.496	19.555
P		<0.001	<0.001	<0.001	<0.001

1 BMD: bone mineral density.

**Table 3:** Associations between BMI^1^ and FRAX-based 10-year osteoporotic fracture probabilities.

		Without BMD^2^		With BMD	
		MOFP^3^	HOFP^4^	MOFP	HOFP
All subjects	r	-0.237	-0.339	-0.113	-0.139
	P	<0.001	<0.001	0.018	0.004
Males	r	-0.238	-0.316	-0.016	-0.042
	P	0.036	0.005	0.887	0.717
Females	r	-0.223	-0.338	-0.105	-0.150
	P	<0.001	<0.001	0.047	0.005

Note: The result was derived based on partial correlation analysis after controlling for age;

1 BMI: body mass index;

2 BMD: bone mineral density;

3 MOFP: FRAX-based 10-year major osteoporotic fracture probability;

4 HOFP: FRAX-based 10-year hip osteoporotic fracture probability.

**Table 4:** FRAX-based 10-year fracture probabilities among groups with different BMD^1^ levels in the risk stratification analysis.

Stratum	Group	Without BMD		With BMD	
		Major fracture	Hip fracture	Major fracture	Hip fracture
Normal BMD based on FN^2^	Normal BMD based on LS^3^	3.36	0.68	2.66	0.23
	Osteopenia based on LS	4.31	0.98	3.14	0.25
	Osteoporosis based on LS	3.34	0.66	2.84	0.3
	ANOVA F statistic	1.75	1.326	1.431	0.827
	P	0.19	0.253	0.235	0.366
Osteopenia based on FN	Normal BMD based on LS	4.51	1.48	4.17	1.13
	Osteopenia based on LS	4.55	1.37	4.24	1.05
	Osteoporosis based on LS	4.87	1.36	4.92	1.24
	ANOVA F statistic	0.435	0.248	3.449	0.419
	P	0.51	0.619	0.065	0.518
Osteoporosis based on FN	Normal BMD based on LS	6.07	2.15	7.7	3.03
	Osteopenia based on LS	6.66	3.04	7.13	3.18
	Osteoporosis based on LS	6.7	2.86	8.46	3.78
	ANOVA F statistic	0.076	0.054	1.045	0.671
	P	0.783	0.816	0.309	0.414
Normal BMD based on LS	Normal BMD based on FN	3.35	0.68	2.66	0.23
	Osteopenia based on FN	4.51	1.48	4.17	1.13
	Osteoporosis based on FN	6.07	2.15	7.7	3.03
	ANOVA F statistic	9.039	16.187	40.152	62.962
	P	0.003	<0.001	<0.001	<0.001
Osteopenia based on LS	Normal BMD based on FN	4.31	0.98	3.14	0.25
	Osteopenia based on FN	4.54	1.37	4.24	1.05
	Osteoporosis based on FN	6.66	3.04	7.13	3.18
	ANOVA F statistic	8.723	23.118	38.424	84.782
	P	0.004	<0.001	<0.001	<0.001
Osteoporosis based on LS	Normal BMD based on FN	3.34	0.66	2.84	0.3
	Osteopenia based on FN	4.87	1.36	4.92	1.23
	Osteoporosis based on FN	6.7	2.86	8.46	3.78
	ANOVA F statistic	10.297	16.249	26.795	27.027
	P	0.002	<0.001	<0.001	<0.001

1 BMD: bone mineral density;

2 FN: femoral neck;

3 LS: lumbar spine.

**Table 5:** Associations between FRAX-based 10-year fracture probabilities and BMD^1^ at different sites.

		Without BMD		With BMD	
		MOFP^2^	HOFP^3^	MOFP	HOFP
FN BMD	r	-0.60	-0.60	-0.34	-0.39
	P	<0.001	<0.001	<0.001	<0.001
	r^4^	-0.52	-0.54	-0.27	-0.34
	P	<0.001	<0.001	<0.001	<0.001
LS BMD	r	-0.21	-0.21	-0.34	-0.30
	P	<0.001	<0.001	<0.001	<0.001
	r^5^	-0.02	0.02	-0.01	0.05
	P	0.615	0.663	0.897	0.265

1 BMD: bone mineral density;

2 MOFP: FRAX-based 10-year major osteoporotic fracture probability;

3 HOFP: FRAX-based 10-year hip osteoporotic fracture probability;

4 the relative coefficient derived based on a partial correlation analysis controlling for LS BMD;

5 the relative coefficient derived based on a partial correlation analysis controlling for FN BMD.
